# Health Status and Quality of Life in the Population near Zhezkazgan Copper Smelter, Kazakhstan

**DOI:** 10.1155/2023/8477964

**Published:** 2023-01-30

**Authors:** Daulet Medgatuly Askarov, Meiram Kaziyevich Amrin, Aigulsum Kulyntayevna Izekenova, Zhanat Bekmukhanbetovna Beisenbinova, Askhat Tursunkhanovich Dosmukhametov

**Affiliations:** ^1^Asfendiyarov Kazakh National Medical University, Tole Bi 94, Almaty 050012, Kazakhstan; ^2^Republican State Enterprise, Research Center “Infrakos”, Abay Avenue 191, Almaty 050046, Kazakhstan; ^3^Kenesary Company LLP, Khadzhimukan 12/2, Almaty 050059, Kazakhstan

## Abstract

**Background:**

The industrial city of Zhezkazgan is one of the most important cities in the industrial sector and the most polluted city in the Republic of Kazakhstan. There is placed Kazakhstan's largest copper smelter. The entire technological process (extraction, crushing, grinding, purification, and smelting of pure ingots) of the production of the copper smelter releases into the environment mainly various kinds of solid particles, sulfur oxides (SOx), and various carcinogenic elements. Emissions from the industrial facilities extend to a significant area around the city, combined with other sources of environmental pollution (motor transport, thermal power plant, individual heating systems, and others).

**Objective:**

This study assessed the health status of residents of villages near Zhezkazgan by screening, quality of life studies, and official medical statistics.

**Methods:**

This study assessed the health status and quality of life of residents near Zhezkazgan city. The cohort included residents from Talap village (main group) and Malshybai village (comparison group) from the Ulytau district in the Karaganda region. The sampling for the health check and quality of life survey covered 260 adult residents of Talap village and 146 adult residents of Malshybai village. Univariate analysis was used to calculate the odds ratio (OR) with a 95% confidence interval (95% CI).

**Results:**

In the city district of Zhezkazgan, the overall mortality rate and mortality from diseases of the circulatory system, neoplasms, and respiratory diseases were much higher than in the Karaganda region and the Republic of Kazakhstan from 2015–2020. Residents of the Talap settlement had higher rates of coronary heart disease (CHD) (OR 1.30; 95% CI: 0.70–2.39; and *p* < 0.05), arterial hypertension (AH) (OR 1.84; 95% CI: 1.11–3.03; and *p* < 0.05), decreased hemoglobin (OR 1.89; 95% CI: 1.17–3.07; and *p* < 0.05), and endocrine diseases (diabetes mellitus, obesity, and thyrotoxicosis) (OR 1.76; 95% CI: 1.12–2.79; and *p* < 0.05) at registration than residents of the Malshybai settlement. Residents of both settlements expressed dissatisfaction with the quality of drinking water and the presence of the area where launch vehicles fell.

**Conclusion:**

Indicators of pollution in the city, statistics of official mortality, and differences in morbidity indicated the negative impact of hazardous emissions from industrial facilities of the copper smelter on public health.

## 1. Introduction

The development of large megacities is largely accompanied by the presence of large industries that emit pollution into the environment, which include copper mining and copper smelting. The largest share of the GDP for the Republic of Kazakhstan (more than 75%) comes from raw materials such as oil and natural gas and metallurgy. Established enterprises in large cities have been a source of anthropogenic environmental pollution since their foundation in the USSR until today.

The habitat of the city of Zhezkazgan and the settlements of adjacent territories are exposed to various types of pollution. One of the main reasons for the unfavorable environmental situation in the region is the copper smelter (the largest in Kazakhstan) and its auxiliary complexes located inside the city (Figure 1). The situation is complicated by outdated technical equipment, which releases large volumes of suspended particles, sulfur oxides, hydrogen sulfide, arsenic, lead, copper, and its compounds into the atmospheric air, as indicated by a risk assessment investigation of air pollution in 2017 [1].

The mining process is accompanied by emissions generated during material handling operations. Copper and iron oxides are the main components of the particulate matter of the mined rocks, but other oxides such as arsenic, antimony, cadmium, lead, Mercury, and zinc may be present, along with metallic sulfates and sulfuric acid mist. Due to the significant amount of sulfur in ores containing copper, considerable sulfur dioxide emissions occur as a result of various processes associated with primary copper smelting. Emissions are also generated as a result of working melting furnaces and converters. Fuel combustion products also contribute to emissions. Analyzing the entire process of mining and smelting, there is pollution in the city with various heavy metals, poisonous gases, and suspended particles.

Official data from the RSE “Kazhydromet” [2] (the state and private enterprises that monitors the state of the environment) for 2018–2021 shows the maximum permissible concentration (MPC_current maximum_ and MPC_daily average_) of pollutants (Kazakhstan normative) was exceeded in Zhezkazgan city [3]. The MPC exceeded at least two-fold for suspended particles (dust), sulfur dioxide, carbon monoxide, nitrogen dioxide, hydrogen sulfide, heavy metals, and phenol. In 2019 and 2021, average annual (MPC_daily average_) concentration of PM_2.5_ were 11–18 *μ*g/m3 and PM_10_ were 18–90 *μ*g/m3, which is higher than air quality guideline level of WHO [4] (PM_2.5_ = 5 *μ*g/m^3^ and PM_10_ = 15 *μ*g/m^3^). Relatively high values were observed for hydrogen sulfide, 7.8–36.6 fold higher than the MPC_current maximum_.

The negative effects of industrial emissions affect people's health in various ways. For example, a scoping review of 799 articles on the impact of outdoor air pollution on health conducted from 1992 to 2008 in various continents showed mainly respiratory diseases (asthma) and mortality (in the medical record) [5]. Research of air pollution in the United States reveals: uncalibrated burden estimates of death due to nonaccidental causes associated with PM_2.5_ from ensembled models for the contiguous United States were 208,500.1 deaths (95% UI, 193,285.2–225,082.6 deaths), 5.4% higher than the Global Exposure Mortality Model–based estimate [6].

There were positive associations between cardiovascular diseases (CVD) and particulate matters (PM) after accounting for competing risk factors: the multivariable-adjusted odds for the multiplicity of CVD outcomes increased by 1.32 (95% CI: 1.23–1.43) and 1.15 (1.07–1.22) times per 10 *μ*g/m_3_ increase in PM_2.5_ and PM_10_, respectively in the latent class regression analyses. [7]. The increased amount of PM, including dust, PM_2.5_, PM_10_, and ozone and nitrogen oxides (dioxides) in the air, leads to relatively higher mortality among the population [8–10].

A second equally important cause of long-term anthropogenic impact that might affect human health is rocket and space activities, which use toxic unsymmetrical dimethylhydrazine (UDMH) or kerosene (T-1) as fuel [11–13]. Over the 65 years that the Baikonur Cosmodrome has been operating, more than 1400 launches have been made, with approximately 7% resulting in accidents. The Baikonur Cosmodrome is located 25 km south of the city of Zhezkazgan, and the surrounding area endures regular rocket stage falls during launches. In addition, the health of the rural population near Zhezkazgan is affected by socio-hygienic factors, such as the harsh climate, poor medical care, and unemployment.

## 2. Methods

For an exhaustive assessment of the possible adverse effects of environmental factors on humans, only laboratory and instrumental studies on environmental pollution are not enough. They should be supplemented by field studies on the population, i.e., epidemiological studies. The main attention in these studies is paid to the study of quantitative relationships between the degree of influence of actually present environmental factors and the state of health of the population, the assessment of the spread of changes in the functional state of the organism in connection with the social and quality of the habitat in urban agglomerations, and on the territories of agro-industrial complexes.

Residents of territories under the administration of the city of Zhezkazgan in the Karaganda region were selected to conduct a health screening study and a quality of life survey. The main group included residents of Talap village (with winter quarters*∗*) and the comparison group included residents of Malshybai village (with winter quarters). Talap village is 12.8 km away to the southeast and Malshybai village is 66 km away to the north of Zhezkazgan (Figure 1). The climatic, ecological, and social conditions of settlements are the same. According to the wind rose, Zhezkazgan has a more frequent north-east wind direction. And Malshybai village, practically, is not affected by emissions from the city [14].

The village of Talap is the closest settlement to Zhezkazgan, where most economically active residents work in the city.

The study was conducted in 2021. According to the Akimats (regional executive bodies of state power) of the studied villages, in 2021, the adult populations of Talap and Malshybai villages were 632 and 414, respectively. Health screening and the quality of life survey covered all existing adult population (18 and older). The coverage was 260 residents of Talap and 146 residents of Malshybai village.

The health screening and questionnaire survey on the quality of life were carried out by the organization approved by the Republican State Enterprise (Infrakos) of the Ministry of Digital Development, Innovations, and Aerospace Industry of the Republic of Kazakhstan. General practitioners from the city of Almaty were involved in medical examinations (Tables1 and 2).

One of the directions of the state policy in the field of public health protection is the preventive orientation of health care. The main form of implementation of this direction is a system of preventive medical examinations of target groups of the population (screening examinations). Screening examinations are designed to detect pathologies at early stages and prevent their further development, including identifying “risk groups” for diseases caused by environmental factors (pollution, psychoemotional state, quality of life, etc.). Modern screening systems are used in many developed countries. According to the recommendations of the World Health Organization, screening examination programs should include both tests for early diagnosis of pathological conditions and identification of risks of developing chronic noncommunicable diseases that can lead to death [15].

Cardiovascular diseases, diseases of the nervous system, mental disorders, neoplasms, pathological conditions during pregnancy, primary morbidity and nontraumatic mortality, nonspecific lung diseases, chronic infections, allergization of the population, and disorders associated with chronic stress can act as an eco-dependent pathology. According to the results of the analysis of the main indicators of population health, significantly lower levels of population and individual health of the population at risk were established in comparison with persons living in conditionally clean settlements.

### 2.1. Screening Study

The “Screening card for adults” contained the following questions:

- Information about the respondent (full name, gender, age, place of residence, labor activity, profession, position, professional experience, presence of hazards, and work experience in hazardous conditions)
- General information (social status, education, marital status, family conflicts, industrial conflicts, bad habits, alcohol tolerance, and drug intolerance)
- Medical status (current complaints and anamnesis vitae)

An objective examination included examination of the skin, oral cavity, and mucous membranes, palpation of superficial lymph nodes, assessment of respiration, gastrointestinal tract, palpation of the liver, neuropsychiatric disorders, and emotional state. Data from laboratory studies and conclusions from outpatient records were interpreted with actual examinations and entered into the patient's screening card.

The quality of life questionnaire consisted of five blocks: (I) physical, (II) psychological, (III) level of independence, (IV) social relationships, (V) environment, and was based on a measurement tool for assessing the quality of life developed by the WHO (WHOQOL-BREF 100) [16]. Questionnaires also reveal the psychoemotional state of residents.

Each question on the quality of life questionnaire was scored on a scale of 1 to 5 (for example, very poor = 1, excellent = 5, or very often = 1, never = 5), and the arithmetic average was calculated. As a result, an integral assessment of the quality of life (Int. AQL) was calculated.

(1) $$\begin{array}{c} \text{Int}.\text{AQL}=\frac{\left(I+\text{II}+\text{III}+\text{IV}+V\right)}{5}\text{.} \end{array}$$

Before the survey, informed consent was taken from the study participants for data analysis. The names of the respondents were filled in with ordinal ciphers.

### 2.2. Statistical Analysis

Univariate analysis was used to calculate the odds ratio for the main (Talap) and comparison (Malshybai) groups with a 95% confidence interval (95% CI).

## 3. Results

The screening survey revealed a similar proportion of men and women in both study groups, with a slightly higher number of women in the main group and a slightly higher number of men in the comparison group. Both study groups had a higher percentage of persons in each of the older age bands (aged 40 and above) than in the younger age bands (aged 18–39).

The majority of the residents of both villages, 85.4% (Talap) and 94.5% (Malshybai), were Kazakhs.

The education level of both villages was similar. Less than 15% of respondents had passed through higher education. Most respondents (82–84%) had a general secondary education or special secondary (postsecondary) level of education.

In terms of employment, there were more unemployed persons in the comparison group (Malshybai) than in Talap (main group).

Similar numbers of respondents in both groups had a disability, 6.8% in the main group (Talap) and 8.8% in the comparison group (Malshybai).

The comparison group (Malshybai) had a slightly higher percentage of smokers than the main group (Talap), 19.2% vs. 13.5%, respectively (Table 3).

### 3.1. Health Screening

During the examination, 14.6% of Talap residents and 10.1% of Malshybai residents were registered at the dispensary for coronary heart disease (CHD) (OR 1.30; 95% CI: 0.70–2.39; and *p* > 0.05). The diagnosis of arterial hypertension (AH) occurred 1.6-fold more often in Talap compared to Malshybai (OR 1.84; 95% CI: 1.11–3.03; and *p* < 0.05).

Nephrological profiling showed that diseases of the kidneys and urinary tract occurred at similar levels in both Talap and Malshybai villages, 25.4% and 23.3%, respectively (OR 1.12; 95% CI: 0.70–1.80; and *p* > 0.05). Gastrological disorders were also present at similar levels in both villages, 40% (Talap) and 43.8% (Malshybai) (OR 0.85; 95% CI: 0.57–1.29; and *p* > 0.05).

Decreased levels of hemoglobin (OR 1.89; 95% CI: 1.17–3.07; and *p* < 0.05) and incidences of endocrine disorders, such as diabetes mellitus, obesity, and thyrotoxicosis (OR 1.76; 95% CI: 1.12–2,79; and *p* < 0.05) were higher in Talap (31.9 and 35.8%, respectively) than that in Malshybai (19.9% and 24.0%, respectively). The percentage of neurological disorders was the same in both villages at 12.3% (OR 0.998; 95% CI: 0.54–1.85; and *p* > 0.05) (see Table 4).

### 3.2. Quality of Life Survey Results

The survey yielded similar results for most questions for both the main group (Talap village) and the comparison group (Malshybai village).

Questions about the environment revealed concern in both the main and comparison groups. Satisfaction with the quality of drinking water was rated as 1.6 and 1.9 for the main and comparison groups, respectively. When residents were asked if they suffered from atmospheric dustiness, scores of 2.9 and 3.0 for the main and comparison groups, respectively, were reported.

The residents of both settlements responded extremely negatively when asked if launches from the Baikonur Cosmodrome affected them (1.1 and 1.6 for the main and comparison groups, respectively).

The integral indicator of the quality of life assessment in Talap village was 4.26 points (out of 5) and 4.16 in Malshybai village (Tables 5 and 6).

## 4. Discussion

The highest level of sulfur dioxide emissions into the atmosphere is explained by the fact that some technological equipment, for example, in the sulfuric acid workshop has been in operation for more than 30 years and the complete utilization of sulfur dioxide in the workshop is not ensured. In addition, with the launch of a new ore-thermal furnace in 2018, the company does not provide complete purification of flue gases from sulfur dioxide.

According to RSE “Kazhydromet,” 15 chemicals are included in the list of priority pollutants in the city of Zhezkazgan. Of the analyzed substances in 2021, 4 substances had carcinogenic properties-cadmium (Cd), chromium (Cr), lead (Pb), and arsenic (As) [2].

According to the risk assessment methodology developed by the United States Environmental Protection Agency (US EPA), excess of these pollutants (acute and chronic exposure) can lead to respiratory diseases, cardiovascular diseases, and diseases of the hematopoietic organs [17, 18].

To assess the social, demographic, and medical well-being of a particular territory, it is necessary to take into account not only birth rates, but also mortality rates. Mortality rates reflect very complex demographic processes. Mortality is influenced by many biological, social, and medical factors. For such comparative studies, mortality rates from cardiovascular diseases, myocardial infarction, and especially malignant neoplasms are used, previously standardizing them by gender and age. These indicators are used in the study of both chronic and acute effects of pollutants. This is especially true of the carcinogenic effect of pollutants. It must be remembered that this characteristic of the state of health should be applied to a sufficient population (at least 10,000).

The Bureau of National Statistics for the Republic of Kazakhstan also indicates that in the city district of Zhezkazgan, the overall mortality rate and mortality from diseases of the circulatory system, neoplasms, and respiratory organs is much higher than in the rest of the region and the republic [19] (Figure 2).

Studies of atmospheric air near a copper smelter in Serbia (Bor) showed above limit values prescribed by EU Directives (1999/30/CE, 2000/105/CE) of heavy metals Pb, Cd, Cu, Ni, and As in PM_10_ [20]. Research data in Gusi City, eastern China (the largest copper smelters in China), revealed high concentrations of Zn (16.02 to 61.48 mg·kg^−1^), Cr (0.23–13.64 mg·kg^−1^), Ni (0.10–5.90 mg·kg^−1^), and Pb (0.15–3.62 mg·kg^−1^) in vegetables with a high hazard index for heavy metal diseases [21]. Urinary samples near a copper smelter in Korea shows decreased cadmium level according to the distance of living. Distance from the smelter was a determinant factor for a decrease of As, Pb, and Cd in multiple regression models [22]. Studies of mortality rates during copper smelter strike in four southeast US states (New Mexico, Arizona, Utah, and Nevada) from 15 July 1967 through the beginning of April 1968, shows that the strike-related estimated percent decrease in mortality was 2.5% (95% CI, 1.1–4.0%) [23]. Risk assessment (Adarsh Kumar et al.) of old copper smelter soil in Karabash (Russia) show high concentrations of Cu, Zn, Pb, As, Cd, and Hg compared with the reference. The author suggests the release of a huge volume of potentially toxic metal (loids) in the environment caused human health issues. The hazard quotient and hazard index were 20 times higher for children and slightly >1 for adults [24]. And another copper smelter emission product (heavy metals) exposure study of risk assessment indicates the same problem [25, 26].

Considering studies near copper smelter plants, we assume that emissions from the metallurgical plant, pollution of the habitat with heavy metals, and other pollutants in Zhezkazgan and nearby settlements with high probability led to frequent registered cases of cardiovascular system (CHD and AH), endocrine system (diabetes mellitus, obesity, and thyrotoxicosis), and hemoglobin disorders in Talap village. The neuropsychological tension of environmental pollution and the presence of rocket launch falling stage area also aggravate the situation and increase the growth of psychosomatic diseases among the population. In addition, the city of Zhezkazgan and nearby settlements in the region have problems with the quality of water supply, irrational nutrition, harsh climate, and other factors that require a more in-depth analysis.

## 5. Conclusion

Analyzing official mortality rates and revealing patterns of the emission impact from copper smelters around the world, showed similarities to the findings in our research, in negative effects on the health of Talap habitats.

Results of the study allow us to conclude that in Talap village (located in the zone of influence for emissions from the industrial facilities of copper smelter), the prevalence of the diseases of cardiovascular system (CHD and AH), endocrine system (diabetes mellitus, obesity, and thyrotoxicosis) and hemoglobin disorders are more common in comparison to the residents of Malshybai village. Most chronic diseases appear to have a connection to decades of anthropological environmental problems that affected Talap village habitats, which can also be linked to Zhezkazgan city.

In addition, the residents of Talap are slightly more dissatisfied with the environment. Attention is drawn to the dissatisfaction of residents with the quality of drinking water and concern about the presence of rocket launch falling stage area near their settlements, even if it is located significantly far away.

People aged over 40 in Talap and over 50 in Malshybai village had a more negative response to health indicators. At a younger age, respondents showed less concern about their health and harmful environmental factors.

In our earlier studies in the habitat of settlements adjacent to the areas of rocket and space activity, chemical contamination of soil, water, and air with rocket fuel and products of its chemical transformation were not detected. At the same time, some residents complain about the deterioration of their health after the launch vehicle crashes. This is evidence that local residents suffer psychoemotional stress associated with the impact of diverse negative environmental factors.

The data obtained indicate that among the population, due to prolonged emotional stress associated with man-made impacts, the risk of cardiovascular diseases, nervous system, sleep disorders, depression, increased excitability or anxiety, as well as other manifestations of psychological impact is increased and worsens their prognosis.

This makes it necessary to conduct in-depth medical examinations and examinations of the neuropsychiatric state of residents. The in-depth program of preventive medical examination provides for the availability of specific individualized recommendations for patients and the prevention of further complications.

In summary, as a result of the analysis, we came to the conclusion that Talap villages and Zhezkazgan city has an unfavorable situation regarding the health and quality of life of the local population.

To find and establish more detailed cause-and-effect relationships in the local ecosystem we need to monitor the content of heavy metals and other chemical elements.

## Figures and Tables

**Figure 1:** The location of Zhezkazgan city, Talap, and Malshybai villages in the Karaganda region (©Yandex map). ^*∗*^winter quarters-structure in the steppe for temporary residence of cattle breeders and shepherds.

**Figure 2:** Mortality rate (by causes) in the city district Zhezkazgan, Karaganda region, and the Republic of Kazakhstan (RK) for 2015–2020 per 100,000 population.

**Table 1:** Screening card for adult.

1. General information
1. Region
2. Date of screening
3. Full name
4. Age
5. Nationality
6. Gender: M-F
7. Monthly income per 1 family member
8. Home address
9. Education: without education, primary, secondary, secondary special, higher
10. Occupation
11. Place of work
12. Position
13. Harmful factors at work: vibration, dust, cooling, physical exertion, etc.
14. Disability from childhood what disease
15. Disabled (which groups 1, 2, 3) what disease
16. Determination date of disability
17. How long did you live in this place (years)
18. Marital status: married, single, widow
19. Smokes: no, yes (<10, >10 cigarettes per day)
20. Consumes alcohol: no, yes, how many: <0.5 liters per week, >0.5 liters per week wine, vodka, beer

II. Anamnesis
Diseases:
1. Measles, mumps, chickenpox, scarlet fever, whooping cough, dysentery, etc.
2. Congenital malformations
3. Травмы (Жарақаттар)-yes, no
4. Seizures with loss of consciousness-yes, no
5. Operations to
6. Venereal diseases, (detection year)
7. Dizziness constantly, often, rarely, no
8. Noise in head constantly, often, rarely, no
9. Heartache constantly, often, rarely, no
10. Dyspnea, suffocation constantly, often, rarely, no
11. Accelerated heartbeat constantly, often, rarely, no
12. Heart failure constantly, often, rarely, no
13 Legs swelling constantly, often, rarely, no
14. Jaundice (detection year)

1. Pulmonological profile
1. Detected lung tuberculosis (detection year)
2. Dispensary observation for non-tuberculosis lung diseases-yes, no
3. Attacks of suffocation-yes, no
4. Cough: persistent, frequent, rare.
5. Frequent bronchitis, pneumonia-yes, no
6. Colds with cough, runny nose currently-yes, no
7. Cough more than 2 months a year.-yes, no
8. Sputum secretion: constantly, often, rarely, no
9. Feeling of wheezing in the chest: constantly, often, rarely, no
10. Chest pain: constantly, often, rarely, no
11. Dyspnea, shortness of breath: constantly, often, rarely, no
12. Elevated temperature: constantly, often, rarely, no
13. Frequent colds: 3–5 times a year, more than 5 times.
14. Allergy-yes, no
15. Operated because of lung diseases-yes, no

2. Cardio rheumatology profile
1. Dispensary observation: for rheumatism, chorea, coronary heart disease, hypertension, etc. -yes, no
2. Had a rheumatism, chorea, coronary heart disease, hypertension, etc., without dispensary observation-yes, no
3. Detected heart defect, a heart murmur-yes, no
4. Joint pain with redness, swelling-yes, no
5. High blood pressure constantly, often, rarely, no
6. Low blood pressure constantly, often, rarely, no
7. Headache constantly, often, rarely, no

3. Nephrological profile
1. Dispensary observation of genitourinary system diseases-yes, no
2. Genitourinary system diseases without dispensary observation-yes, no
3. Renal colic-yes, no
4. Urine with blood-yes, no
5. Abnormalities in urine tests-yes, no
6. Painful, difficult urination constantly, often, rarely, no
7. Cloudy urine constantly, often, rarely, no
8. Operated due to kidney and urinary tract disease-yes, no
9. Urinary incontinence-yes, no

4. Gastroenterological profile
1 Observation about hepatitis, pancreatitis, peptic ulcer, other digestive diseases-yes, no
2 Jaundice-no, 1 time, more than 1 time
3. Found stomach ulcer, duodenal ulcer-yes, no
4. Gallstones-yes, no
5. Polyp of the stomach, intestines-yes, no
6. Found worms, giardia-yes, no
7. Increased acidity of gastric juice-yes, no
8. Pain “in the pit of the stomach” constantly, often, rarely, no
9. Pain in the right hypochondrium constantly, often, rarely, no
10. Pains all over the abdomen constantly, often, rarely, no
11. Abdominal pain to empty stomach at night constantly, often, rarely, no
12. Abdominal pain after eating fatty, fried, spicy food constantly, often, rarely, no
13. Seasonality of pain (spring, autumn) constantly, often, rarely, no

5. Hematological profile
1. Dispensary observation about blood diseases-yes, no
2. Decreased hemoglobin, anemia in past-yes, no
3. Bleeding (nasal, hemorrhoidal, other) often, rarely, no
4. Copious menstrual blood loss-yes, no
5. Frequent “bruises,” hemorrhages on the skin-yes, no
6. Found abnormalities in blood tests before constantly, often, rarely, no
7. General weakness constantly, often, rarely, no
8. Admixture of blood in feces-yes, no

6. Endocrinological profile
1. Diagnosed with diabetes mellitus, obesity, thyrotoxicosis-yes, no
2. Other diseases of the endocrine system-yes, no
3. Previously registered an increased sugar in the blood, sugar in the urine-yes, no
4. Loosening, loss of teeth-yes, no
5. Furunculosis, frequent pustular skin diseases-yes, no
6. Thirst constantly, often, rarely, no
7. Weight loss by 4-5 kg over the last year-yes, no
8. Thyroid surgery-yes, no

7. Gynecological profile
1. Pregnancy (how many)
2. Childbirth (how many)
3. Protected-yes, no
4. Was she ill with colpitis, metritis, endocervicitis, inflammation of the uterine appendages-yes, no
5. Uterine tumors-yes, no
6. Ovarian tumors-yes, no
7. Menstrual cycle determined: immediately; after several menstruations; not determined
8. Painful menstruation-yes, no
9. Undergone surgery on the genitals (removal of the uterus, appendages, cesarean section, ectopic pregnancy, etc.)–yes, no

8. Nervous diseases
1. Dispensary observation by a neurologist: no; yes
2. Complaints of headache: no; dull diffusion, paroxysmal.
3. Headache rarely, periodically, constantly
4. Headache is accompanied by nausea, vomiting-yes, no
5. Loss of consciousness-yes, no
6. Convulsions Судороги: no; generalized; local; small; febrile
7. Dizziness-yes, no
8. Nystagmus-yes, no
9. Muscle strength: preserved; reduced
10. Sensitivity: reserved, broken superficially; deeply
11. Sleep: not disturbed; disturbed
12. Speech is impaired: no; stuttering; dysarthria (violation of the pronunciation side of speech); aphasia (loss of the ability to use words and phrases as a means of expressing thoughts).
13. Memory impairment: none; reduced.
14. Memory decline expressed, unexpressed, none

9. Additional information
1. Irritable, calm
2. The ability to have sexual relations-preserved, reduced, lost
3. The ability to work-preserved, reduced, lost
4. Fatigue-yes, no
5. Insomnia-yes, no
10. Self-assessment of condition
Assessment on a five-point system
**1 2 3 4 5**
The survey was conducted by ______________________________________ Position, Full name, date

**Table 2:** Questionnaire of quality of life.

1. Gender: Male, female
2. Age:
3. Nationality:
4. Duration of residence in the locality: -less than 5, 5–9 years, 10–19 years, 20 and more year
5. Education: incomplete secondary, secondary, specialized secondary, incomplete higher, higher
6. Marital status: married, divorced, widower, single
7. Occupation: worker, government worker, farmer, pensioner, student, housewife, individual work activity, unemployed
8. Disability (Group): 1, 2, 3
9. Frequency of visits to healthcare facilities during the year Not once. [5], 1–4 times [4], 5–9 times [3], monthly [2], weekly [1]
10. How often do respiratory diseases signs (runny nose, sneezing, cough, etc.) occur during the year Not once. [5], 1–4 times [4], 5–9 times [3], monthly [2], weekly [1]
11. How often do signs of the stomach, intestinal diseases, diarrhea, nausea, vomiting, etc. occur during the year Not once. [5], 1–4 times [4], 5–9 times [3], monthly [2], weekly [1]
12. How often do signs of heart and vascular disease (heart pain, swelling, increased blood pressure, etc.) occur during the year Not once. [5], 1–4 times [4], 5–9 times [3], monthly [2], weekly [1]
13. How often do skin changes (itching, redness, enlarged lymph nodes, etc.) occur during the year Not once. [5], 1–4 times [4], 5–9 times [3], monthly [2], weekly [1]
14. How often do signs of kidney disease (frequent and difficult urination, etc.) occur during the year Not once. [5], 1–4 times [4], 5–9 times [3], monthly [2], weekly [1]
15. How often do signs of nervous diseases (irritability, insomnia, spinal pain, etc.) occur during the year Not once. [5], 1–4 times [4], 5–9 times [3], monthly [2], weekly [1]
16. How often do you experience pain: do not [5], relatively rarely [4], relatively often [3], often [2], very often [1]
17. Are you worried about physical pain or discomfort? No [5], a little [4], moderately [3], relatively strongly [2], Very strongly [1]
18. Do you have enough energy for everyday life? Yes [5], a little lacking [4], moderately lacking [3], severely lacking [2], very much lacking [1]
19. How easily do you get tired? No [5], relatively rarely [4], moderately [3], strongly [2], very strongly [1]
20. How well do you sleep? Very good [5], good [4], satisfactory [3], Bad [2], Very bad [1].
21 How do you assess your health now? Very good [5], good [4], satisfactory [3], Bad [2], Very Bad [1].
22. Emotional state during the last 4 weeks caused difficulties at work, in communicating with family, relatives, neighbors or work colleagues: No [5]; a little [4]; moderately [3]; strongly [2]; Very strongly [1].
23. Your mood during the last 4 weeks. Did you feel cheerful and calm: Very often [5]; often [4]; sometimes [3]; rarely [2]; never [1].
24. Your mood during the last 4 weeks. Were you nervous and feeling depressed? Never [5] rarely [4] sometimes [3]; often [2]; very often [1]
25. Do family and household conflicts often occur? Very rarely [5]; rarely [4], sometimes [3]; often [2]; very often [1].
26. How satisfied are you with your ability to learn new things, focus attention and make decisions? Very strongly [5]; strongly [4], moderately [3]; little [2]; not satisfied [1].
27. How satisfied are you with your appearance and yourself? Very strongly [5]; strongly [4], moderately [3]; little [2]; not satisfied [1].
28. How well are you able to move around? Very good [5], good [4], satisfactory [3], bad [2], very bad [1].
29. To what extent are you able to cope with everyday tasks? Very good [5], good [4], satisfactory [3], bad [2], very bad [1].
30. Are you dependent on medications? No [5]; a little [4]; moderately [3]; strongly [2]; very strongly [1].
31. How badly do you need any medical treatment for everyday life? No [5], a little [4], moderately [3], relatively strongly [2], Very strongly [1]
32. Can you work? Fully [5]; slightly less [4], moderately less [3], little [2], not at all [1]
33. Personal relationships with relatives, friends, neighbors and colleagues Very good [5], good [4], satisfactory [3], bad [2], very bad [1].
34. Do you feel happy in communicating with your family members? Fully [5]; slightly less [4], moderately less [3], little [2], not at all [1]
35. Do you get any support from others when you need it? Fully [5]; slightly less [4], moderately less [3], little [2], not at all [1]
36. How satisfied are you with the support you receive from others? Fully [5]; slightly less [4], moderately less [3], little [2], not at all [1]
37. How safe do you feel in your daily life? Fully [5]; slightly less [4], moderately less [3], little [2], not at all [1]
38. How comfortable is your accommodation (place of residence)? Fully [5]; slightly less [4], moderately less [3], little comfortable [2], uncomfortable [1].
39. Are you satisfied with your financial situation? Fully [5]; slightly less [4], moderately less [3], little satisfied [2], no [1].
40. How easily can you get qualified medical care? Easy [5]; a little harder [4], moderately harder [3], with great difficulty [2], cannot [1].
41. How satisfied are you with the availability of medical care for you? Fully [5]; slightly less [4], moderately less [3], little satisfied [2], no [1].
42. Are you having trouble in purchasing medicines? No [5], a little [4], moderately [3], relatively strongly [2], Very strongly [1]
43. How do you assess the quality of social assistance available to you? Very good [5], good [4], satisfactory [3], Bad [2], Very bad [1].
44. How accessible is the information you need in your daily life? Fully [5]; slightly less [4], moderately less [3], little available [2], not available [1].
45. What are the opportunities for recreation and entertainment? Very good [5], good [4], satisfactory [3], Bad [2], Very bad [1].
46. How important is the adequate operation of transport in everyday life for you? Fully [5]; slightly less [4], moderately less [3], Little important [2], not important [1].
47. Do you smoke? (How much) No [5]; 1–3 cigarettes per day [4]; up to 0.5 packs per day [3]; up to a pack per day [2]; more than one pack per day [1].
48. Alcohol consumption No [5], on holidays [4], once a month [3], once a week [2]; every day [1].
49. Drug use (Есірткіні пайдалану) yes [1], No [5]
50. Do you suffer from dustiness of the atmospheric air? No [5], slightly [4], moderately [3], strongly [2], very strongly [1]
51. Are you satisfied with the climate? Fully [5]; slightly less [4], moderately [3], little [2], no [1]
52. Are you satisfied with the quality of drinking water? (Ауыз судың сапасы қанағаттандыра ма?) Fully [5]; slightly less [4], moderately [3], little [2], no [1]
53. Are you satisfied with the landscaping of the territory? Fully [5]; slightly less [4], moderately [3], little [2], no [1]
54. Are you satisfied with the environment? Fully [5]; slightly less [4], moderately [3], little [2], no [1]
55. Are you concerned about the presence of a cosmodrome in your region, areas of falling of separating parts of launch vehicles? No [5], slightly [4], moderately [3], strongly [2], very strongly [1]
56. Do the launches of launch vehicles from the baikonur cosmodrome affect you? No [5], slightly [4], moderately [3], strongly [2], very strongly [1]
57. The impact effects on the state of health is (underline) environmental pollution; poor drinking water; polluted air; poor living conditions; lack of work; lack of money, poor-quality medical care; conflicts in the family, conflicts at work
58. What needs to be improved in the first place: medical care; job creation; water supply, living conditions, etc.___________________________________

**Table 3:** General information about the surveyed residents of the villages of Talap (main group) and Malshybai (comparison group) with winter quarters in the Ulytau district of the Karaganda region.

		Main group (Talap village)	Comparison group (Malshybai village)
Sample		260	146
	Women, *n* (%)	141 (54.2)	67 (45.9)
	Men, *n* (%)	119 (45.8)	79 (54.1)
Age, *n* (%)	18–29	49 (18.8)	16 (11.0)
	30–39	29 (11.2)	17 (11.6)
	40–49	51 (19.6)	38 (26.0)
	50–59	60 (23.1)	39 (26.7)
	60 and above	71 (27.3)	36 (24.7)
Ethnic group	Kazakh	222 (85.4)	138 (94.5)
	Russian	31 (11.9)	6 (4.1)
	Other	7 (2.7)	2 (1.4)
Employment status, *n* (%)	Unemployed	13 (5.0)	17 (11.6)
	Housewife	7 (2.7)	13 (8.9)
	Pensioner	50 (19.2)	24 (16.4)
	Self-employed	10 (3.8)	20 (13.7)
	Governmental employee	53 (20.4)	16 (11.0)
	Student	4 (1.5)	
	Employed and other types of work	123 (47.3)	56 (38.4)
Education, (%)	No education	1.2	3.5
	Primary	0.4	0.7
	General secondary education	28.5	58.7
	Special secondary	55.9	23.8
	Higher	14.1	13.3
Disability, *n* (%)		23 (8.8)	10 (6.8)
Smokers, *n* (%)		35 (13.5)	28 (19.2)

**Table 4:** Pathologies and symptoms among residents of the villages of Talap (main group) and Malshybai (comparison group) with winter quarters in the Karaganda region.

	Main group (Talap village)	Comparison group (Malshybai village)	Univariate analyses			
			Odds ratio	Lower limit	Upper limit	*P* value
Sample	260	146				
Frequent colds, 3–5 times per year, *n* (%)	35 (13.5)	50 (34.2)	0.299	0.1823	0.4893	<0.05
Allergies	20 (7.7)	28 (19.2)	0.351	0.1899	0.6494	<0.05
Registered CHD	38 (14.6)	17 (10.1)	1.299	0.7046	2.3945	>0.05
Registered AH	74 (28.5)	26 (17.8)	1.836	1.1111	3.0345	<0.05
Diseases of the kidneys and urinary tract without dispensary registration	66 (25.4)	34 (23.3)	1.121	0.6972	1.8014	>0.05
Hepatitis, pancreatitis, peptic ulcers or other digestive obstructions (observed by a doctor)	104 (40.0)	64 (43.8)	0.854	0.5666	1.2876	>0.05
Decreased hemoglobin, previous anemia	83 (31.9)	29 (19.9)	1.892	1.1672	3.0666	<0.05
Diabetes mellitus, obesity, thyrotoxicosis (already diagnosed)	93 (35.8)	35 (24.0)	1.766	1.1185	2.7888	<0.05
Neurological disorders (observed by a neurologist)	32 (12.3)	18 (12.3)	0.998	0.5387	1.8492	>0.05

**Table 5:** Assessment of the quality of life using a five-point scale for the villages of Talap (main group) and Malshybai (comparison group) in the Ulytau district of Karaganda region.

	Main group (Talap village)	Comparison group (Malshybai village)
Frequency of visits to healthcare facilities during the year	4.5	4.4
The frequency of signs of respiratory diseases (runny nose, sneezing, coughing, etc.) during the year	4.6	4.7
The frequency of signs of heart and vascular disease (pain in the heart, swelling, high blood pressure, etc.) per year	4.1	4.3
The frequency of signs of nervous diseases (irritability, insomnia, pain in the spine, etc.) per year	4.5	4.5
How do you rate your health at the moment?	3.8	3.8
How satisfied are you with your access to health care?	3.9	3.9
Do you suffer from air pollution?	2.9	3.0
Are you satisfied with the quality of drinking water?	1.6	1.9
Satisfaction with the financial situation	4.6	4.5
Do the launches of launch vehicles from the baikonur cosmodrome affect you?	1.1	1.6
Average Int. AQL	**4.26**	**4.16**

**Table 6:** Results of the questionnaire for assessing the quality of life in Talap and Malshybai with winter quarters in Ulytau district of Karaganda region.

Points	Main group (Talap village, with winter quarters)					Comparison group (Malshybai village, with winter quarters)				
	**5**	**4**	**3**	**2**	**1**	**5**	**4**	**3**	**2**	**1**
Frequency of visits to healthcare facilities during the year	138	97	9	2	1	65	74	3	3	1
The frequency of signs of respiratory diseases (runny nose, sneezing, coughing, etc.) during the year	144	99	1	0	0	100	40	3	0	0
The frequency of signs of heart and vascular disease (pain in the heart, swelling, high blood pressure, etc.) per year	91	97	57	0	0	70	45	25	1	2
The frequency of signs of nervous diseases (irritability, insomnia, pain in the spine, etc.) per year	153	62	30	0	0	96	31	15	0	1
How do you rate your health at the moment?	74	55	104	12	0	42	36	55	7	0
How satisfied are you with your access to health care?	61	116	57	11	0	32	61	35	6	0
Do you suffer from air pollution?	4	68	111	29	33	8	38	52	15	18
Are you satisfied with the quality of drinking water?	4	37	0	14	190	12	22	2	6	89
Satisfaction with the financial situation	177	43	13	12	0	98	24	9	7	0
Do the launches of launch vehicles from the baikonur cosmodrome affect you?	0	0	0	31	214	10	1	4	25	91

Note: abs. numbers; gradation of points: 5-excellent, 1-very bad.

## Data Availability

Official data of the monitoring pollution in Zhezkazgan city could be found at https://www.kazhydromet.kz/en/ and the overall mortality rate and mortality from diseases in Kazakhstan, regions, and city district of Zhezkazgan in https://stat.gov.kz/region/256619/statistical_information/publication. Other original research data will be available upon request to the authors of the manuscript (Askarov Daulet at askarovdauletmed@gmail.com or Amrin Meiram at meiramamrin308@gmail.com).

## Additional Points

*Study Limitations*. The quality of life questionnaire is subjective. The answers may differ due to the emotional state of the respondent or their dissatisfaction with governing bodies. *Recommendations*. It is necessary to modernize the technological equipment to improve purification and filtration of exhaust emissions and control the implementation of short-term emission reductions during periods of adverse weather conditions, which leads to multiple exceedances of the MPC in the air.

## References

[1] Kenessary D., Kenessary A., Adilgireiuly Z. (2019). Air pollution in Kazakhstan and its health risk assessment. *Annals of Global Health*.

[2] Kazhydromet (2018). *Information Bulletin on the State of the Environment of the Republic of Kazakhstan*.

[3] Kuantyrov A. (2015). Order of the minister of national economy of the republic of Kazakhstan. *Approval of Hygienic Standards for Atmospheric Air in Urban and Rural Settlements*.

[4] Organization W. H. (2021). *WHO global air quality guidelines: particulate matter (PM2.5 and PM10), ozone, nitrogen dioxide, sulfur dioxide and carbon monoxide*.

[5] Sun Z., Zhu D. (2019). Exposure to outdoor air pollution and its human health outcomes: a scoping review. *PLoS One*.

[6] Bowe B., Xie Y., Yan Y., Al-Aly Z. (2019). Burden of cause-specific mortality associated with PM2.5 air pollution in the United States. *JAMA Network Open*.

[7] Feng J., Yang W. (2012). Effects of particulate air pollution on cardiovascular health: a population health risk assessment. *PLoS One*.

[8] Di Q., Wang Y., Zanobetti A. (2017). Air pollution and mortality in the medicare population. *New England Journal of Medicine*.

[9] Stafoggia M., Oftedal B., Chen J. (2022). Long-term exposure to low ambient air pollution concentrations and mortality among 28 million people: results from seven large European cohorts within the ELAPSE project. *The Lancet Planetary Health*.

[10] Kasdagli M. I., Katsouyanni K., de Hoogh K., Lagiou P., Samoli E. (2022). Investigating the association between long-term exposure to air pollution and greenness with mortality from neurological, cardio-metabolic and chronic obstructive pulmonary diseases in Greece. *Environmental Pollution*.

[11] Nechaykina O. V., Laptev D. S., Petunov S. G., Bobkov D. V. (2022). Effect of unsymmetrical dimethylhydrazine on isolated heart and lymphatic vessels. *Bulletin of Experimental Biology and Medicine*.

[12] Umitzhanov M., Musaeva A. K., Abishov A. A. (2021). Examination of organs and tissues of adult sheep grazed in an area with possible intoxication with rocket fue, Kazakhstan. *Veterinaria Italiana*.

[13] Council N. R. (2016). *Acute Exposure Guideline Levels for Selected Airborne Chemicals*.

[14] (2022). *The «meteoblue» Climate Diagrams for 30 Years of Hourly Weather Model*.

[15] WHO (2020). *Screening Programmes:a Short Guide. Increase Effectiveness, Maximize Benefits and Minimize Harm*.

[16] World Health Organization Quality of Life (Whoqol) (2012). *User Manual, in Programme On Mental Health*.

[17] Lorber M. (2001). Indirect exposure assessment at the United States environmental protection agency. *Toxicology and Industrial Health*.

[18] Suter G. W. (2008). Ecological risk assessment in the United States environmental protection agency: a historical overview. *Integrated Environmental Assessment and Management*.

[19] (2020). *Statistical Collection of the Demographic Yearbook of the Karaganda Region 2013-2020*.

[20] Nikolić D., Milosevic N., Mihajlovic I. (2010). Multi-criteria analysis of air pollution with SO(2) and PM(10) in urban area around the copper smelter in bor, Serbia. *Water, Air, and Soil Pollution*.

[21] Hu Y., Zhou J., Du B. (2019). Health risks to local residents from the exposure of heavy metals around the largest copper smelter in China. *Ecotoxicology and Environmental Safety*.

[22] Kim Y. D., Eom S. Y., Yim D. H. (2016). Environmental exposure to arsenic, lead, and cadmium in people living near janghang copper smelter in Korea. *Journal of Korean Medical Science*.

[23] Pope C. A., Rodermund D. L., Gee M. M. (2007). Mortality effects of a copper smelter strike and reduced ambient sulfate particulate matter air pollution. *Environmental Health Perspectives*.

[24] Kumar A., Maleva M., Kiseleva I., Maiti S. K., Morozova M. (2020). Toxic metal(loid)s contamination and potential human health risk assessment in the vicinity of century-old copper smelter, Karabash, Russia. *Environmental Geochemistry and Health*.

[25] Du B., Zhou J., Lu B. (2020). Environmental and human health risks from cadmium exposure near an active lead-zinc mine and a copper smelter, China. *Science of The Total Environment*.

[26] Cai L. M., Wang Q. S., Luo J. (2019). Heavy metal contamination and health risk assessment for children near a large Cu-smelter in central China. *Science of the Total Environment*.

